The article "Somatostatin Derivative (smsDX) Targets Cellular Metabolism in Prostate Cancer Cells after Androgen Deprivation Therapy" was retracted in 2024. Reasons: false authorship; a false affiliation; original data or images not available; concerns about the images.

# Somatostatin Derivative (smsDX) Targets Cellular Metabolism in Prostate Cancer Cells after Androgen Deprivation Therapy

**DOI:** 10.1371/journal.pone.0055790

**Published:** 2013-02-07

**Authors:** Lei Yan, Zhaoquan Xing, Zhaoxin Guo, Zhiqing Fang, Wei Jiao, Xiaoyu Guo, Zhonghua Xu, Zhenghui Fang, Zhaoxu Liu

**Affiliations:** 1 Department of Urology, Qilu Hospital, Shandong University, Jinan, China; 2 Aging and Health Center, School of Nursing, Shandong University, Jinan, China; 3 Department of Obstetrics and Gynecology, Jinan Central Hospital, Shandong University, Jinan, China; Queensland University of Technology, Australia

## Abstract

Cancer cell metabolism responsive to androgen deprivation therapy (ADT) may be involved in the development and progression of prostate cancer and the ultimate failure of androgen-deprivation therapy. To investigate the metabolism regulation effects on androgen-independent growth of prostate cancer, an established LNCaP-s cell model that resembles the clinical scenario of castration-resistant prostate cancer (CRPC), was used in this current study. This cell line was cultured from androgen-sensitive LNCaP parental cells, in an androgen-reduced condition, resembling clinical androgen deprivation therapy. To assess the effects of smsDX on the invasiveness of prostate cancer cells we used wound healing assay and Matrigel™ invasion assay. We evaluated differentially expressed proteins of the parental LNCaP cells and LNCaP-s cells after ADT by means of two-dimensional gel electrophoresis (2-DE) followed by MALDI-TOF mass spectrometric analysis. The covered area in the wound and the number of cells invading through a Matrigel chamber were significantly smaller for cells treated with smsDX than they were for control cells treated with vehicle. 56 proteins were found differentially expressed in LNCaP-s cells compared to LNCaP cells, majority of them were down-regulated after ADT treatment. 104 proteins of LNCaP cells and 86 in LNCaP-s cells, separately, were found differentially expressed after treatment with smsDX, When we explored these protein functions within the website UniProtKB/Swiss-Prot, surprisingly, most of the proteins were found to be involved in the cellular metabolism and mitochondrial function regulation. LNCaP-s as potential metastatic androgen-independent cancer cells, its metabolism and mitochondrial functions could be altered by a new somatostatin derivative smsDX, the smsDX regulatory effects on metabolism in LNCaP-s deliver more therapeutic information with the treatment of CRPC.

## Introduction

Prostate cancer is the most common malignancy in men, and the leading cause of cancer-related mortality in US and Europe males [1]. The tumor progression to CRPC stage is a complex process that may be involving both clonal selection and adaptive mechanisms in heterogeneous tumors composed of cells that respond differently to androgen deprivation therapy (ADT). However, the mechanisms by which tumors acquire androgen independence remain unclear and need to be addressed before effective treatment strategies can be developed.

ADT is commonly employed in the treatment of advanced prostate cancer. But androgen deprivation therapy is not curative [2], so the lethal CRPC is inevitable. Signs of vascular degeneration, hypoxia, and metabolic stress in the prostate tumor tissue are exacerbated following surgical or medical castration [3]. After a short remission period, the majority of prostate cancer becomes androgen-independent. CRPC cells after ADT are able to survive the low oxygen and nutrient environment and emerge with a different phenotype. Androgen deprivation is known to induce neuroendocrine (NE) differentiation in LNCaP cells, and involves in the transition to androgen independence [4], [5]. NE tumors have been proven to overexpress somatostatin receptors (SSTRs) [6]. The SSTR1-5 expression could be regulated by somatostatin and its derivative smsDX possible via the regulation of the mitochondria of LNCaP that eventually could trigger mitochondrial-mediated apoptosis [7]. Somatostatin analogs bind to SSTRs and are believed to have dual antitumor activity, both direct (anti-proliferative) and indirect (inhibition of various peptide hormones secreted by the tumor cells) [8], [9]. Somatostatin analog, lanreotide has been demonstrated to have considerable antineoplastic effect in various tumors, including CRPC [10]. But the regulation of somatostatin analog on prostate cancer cellular metabolism has not been clearly addressed.

We argue that inhibition of androgen receptor (AR) expression is in itself sufficient to induce cell death in AR-positive cells. But when these AR-positive cells gradually lost AR expression or in a lower AR expression in prostate cancer cells, those CRPC cells could get energy supply via mitochondrial activities. According to the findings of Sotgia F group [11], epithelial cancer cells could take up energy-rich metabolites from neighboring stromal fibroblasts which provide the necessary energy-rich microenvironment for facilitating tumor growth and angiogenesis. These starved cells stripped of androgen could use these metabolites in the mitochondrial tricarboxylic acid cycle (TCA), resulting in a higher proliferative capacity. For CRPC cells emerging after ADT, up-regulate enzymes that convert adrenal androgens to testosterone and DHT (in particular AKR1C3) further enhancing their intratumoral androgen synthesis and reactivating AR transcriptional activity [12], AR reactivation is increased intratumoral synthesis of testosterone and DHT from weak androgens produced by the possibly *de novo* from cholesterol in host stroma and extracellular metabolites.

The principal problem arising from prostate cancer is its propensity to metastasize. Local invasion is one of the fundamental early steps in metastasis, as without it tumor spread cannot occur. The multistep process of invasion and metastasis has been schematized as a sequence of discrete steps, often termed the invasion-metastasis cascade [13], [14]. During this cascade the metabolic reprogramming to support synthesis of the new proteins, lipids, and nucleic acids is critical for cell growth and division [15]. We speculate that the cellular metabolic alterations would accompany the prostate cancer progress to lethal CRPC status. Our study will focus on the smsDX inhibitory effects on the invasiveness of prostate cancer and regulation of relating cellular metabolism after inhibition of AR activity, mediated by androgen depletion. Using LNCaP and LNCaP-s cells to examine the proteins involving in the cell metabolism and energy functions in prostate cancer and to determine the regulatory effects caused by somatostatin derivative smsDX, we demonstrated ADT down-regulates most of mitochondrial proteins, possibly results in the activation of mitochondrial-mediated apoptotic pathway. The smsDX effects on ER leads to overexpression of GRP78, together with other two ER proteins PDIA1 and PDIA3. smsDX exerts its effects by dysregulating of metabolic enzymes at multiple levels, which involves in the process of CRPC cell invasiveness and survival. In conclusion, these results suggest that ADT regulates mitochondrial-mediated and ER stress signalling in LNCaP cells and leads to reprogramming of metabolism in CRPC cells, smsDX regulatory effects on the CRPC cells provides useful information for the treatment of CRPC.

## Materials and Methods

### Cell culture and Reagents

LNCaP human prostate cancer cell line (American Type Culture Collection, Rockville, MD, USA) were routinely maintained in the regular medium (Phenol Red-positive RPMI 1640 medium supplemented with 5% FBS, 1% glutamine, and 0.5% gentamicin) as described previously at 37°C in a humidified atmosphere of 5% CO_2_. The medium was changed two times by week and the cells were trypsinized and subcultivated once a week. For experiments, androgen sensitive LNCaP cells with passage numbers 28–33 were utilized. To establish an androgen-independent prostate cancer cell line, we cultured a LNCaP-s cell line from a parental prostate cancer cell line LNCaP in a androgen-deprivation condition. After 8–12 passages, LNCaP-s cells were treated with smsDX. Somatostatin was from Ferring, Kiel, Germany. The cell culture was treated with smsDX (from Professor Sten Nilsson Lab) or with somatostatin for three days, 1 nM per day, as described by Liu Z [7]. Anti-human AR, CgA and NSE, anti-TOM40 antibody (sc11414), β-actin (rabbit anti-actin antibody R-22) were purchased from Santa Cruz Biotecnology. TCTP (#5128), STMN1 (#3352) and VDAC2 (#9412) antibodies were purchased from Cell Signaling commercially. CBX3 (HPA004902) and GRP78 (G9043) antibodies were purchased from Sigma commercially.

### Wound healing assay

Cells were grown to confluence on 6-well tissue culture plates and a wound was made by scraping in the middle of the cell monolayer with a P200 pipette tip. After floating cells were removed by extensive washing with ice-cold phosphate buffered saline fresh complete medium containing 10 nM smsDX or the corresponding amount of PBS was added. Migration and cell movement throughout the wound area were examined after 24 hours.

### Matrigel Invasion Assay

Invasion assay was performed using Matrigel coated Transwell inserts (BD™) with 8 µm pores in 24-well plates, as per manufacturer's instructions. Briefly, a suspension of 1×10^6^ cells in 100 µl serum-free medium was added to the insert and 500 µl of RPMI 1640 medium containing 20% FBS supplemented with 1–10 nM smsDX or the corresponding amount of saline were added to the bottom of the well. After the plates were incubated for 48 hours at 37°C the inserts were fixed in methanol, the filters were stained with 0.1% crystal violet and the number of cells that invaded through the Matrigel coated Transwell inserts were counted at 40× magnification. The number of cells was counted in independent triplicate experiments in at least 10 fields per well. The assays were repeated 3 times.

### Western blot analysis

In androgen-dependent LNCaP cells after ADT treatment, we cultured a stable LNCaP-s cell line. The androgen independent prostate cancer cell biomarkers and proteins affected by smsDX were tested. Western blotting was performed to validate several selected differentially expressed proteins identified by 2-DE based MS. Primary antibodies were used at the following dilutions: goat anti-human AR, CgA and NSE, 1∶1000; β-actin, 1∶1500; anti-TOM40 antibody, 1∶800. TCTP, 1∶1000; STMN1, 1∶1000; VDAC2, 1∶1000; CBX3, 1∶1000; GRP78, 1∶1000. Western blots were performed as described [16]. In short, cells were lysed with buffer containing 50 mM Tris-HCl (pH 7.5), 250 mM NaCl, 0.1% NP-40 and 5 mM EGTA, 50 mM sodium flu-oride, 60 mM β-glycerol-phosphate, 0.5 mM sodium-vanadate, 0.1 mM PMSF, 10 µg/ml aprotinin and 10 µg/ml leupeptin. Protein samples (35 µg) were subjected to a 10% SDS-PAGE and electrophoretically transferred to PVDF membranes (Bio-Rad, Hercules, CA, USA). The membranes were first incubated with 5% nonfat milk in Tris-buffered saline (TBS). After washing three times in 0.1% Tween 20-TBS (TBST), the membranes were incubated with different primary antibodies separately at 4°C overnight, followed with the corresponding secondary antibodies separately (1∶2000) for 1 h at room temperature and the antibody-bound proteins were detected by the ECL system (Amersham Biosciences, Little Chalfont Buckinghamshire, UK).

### Sample preparation and protein extraction and concentration

The cellular extraction from LNCaP and LNCaP-s cells and the preparation of the total cell lysate were performed as previously described by [17]. Protein determination was made using Pierce BCA protein assay reagent (Rockford, IL, U.S.A.).

### IEF and SDS-PAGE

The samples were diluted to a total volume of 250 µl, 0.2% Pharmalyte, 8 M urea, 0.3% DTT, 2 M CHAPS and a trace of bromphenol blue (Sigma). An amount of 100 µg of protein was loaded on each strip via rehydration using non-linear pH 3–10 Ready Strip IPG, strips (Bio-Rad, Hercules, Ca, USA). Focusing was carried out for a total of 45,500 Vh in a PROTEAN IEF cell (Bio-Rad). Precast gels (12.5% homogenous Tris-HCL Criterion) SDS-PAGE (Bio-Rad) were run using a Criterion Dodeca cell gel apparatus (Bio-Rad). A total of 4 gels were run per sample group. The electrode running buffer was 25 mM Tris, 192 mM Glycine, 0.1% w/v SDS. Gels were run at 250 V for approximately 1 hour until the bromophenol blue marker had reached the bottom of the gel at a temperature of approximately 15°C. Proteins were visualized by silver staining as described by [18].

### Gel scanning and image analysis

2-DE gels were scanned at 100 µm resolution (12-bits/pixel) using a GS-710 laser densitometer (Bio-Rad). Data was analyzed using PDQuest™ software Version 7 (Bio-Rad). After auto-detection of all protein spots, gel-images were carefully edited. The individual proteins quantities were expressed as ppm of the total integrated OD. All 2-DE maps were matched and evaluated independently. The methodological reproducibility of the 2-DE analysis was determined using group correlation analysis. Briefly, the total optical density is directly correlated to the total protein concentration. Minor differences in gel loading, running conditions, and silver staining may affect sample comparisons and affecting the 2-D gel reproducibility. Four gels were run from each treatment group and comparisons of the intensity of matched spots between 2-DE gels were performed using the correlation coefficient analysis. A correlation coefficient was measured between two gels based on the optical densities of the same spots in the two gels being compared. A correlation coefficient of 1 will imply that the two samples being compared are identical. In a group consisting of 4 samples, a maximum of six pair wise comparisons are possible. The average correlation coefficient among the smsDX samples was 0.85 (n = 6 gel pairs, range 0.80–0.92).

### Mass spectrometry analysis

Proteins were identified with a vMALDI-LTQ instrument (Thermo Electron, San José, CA, USA). The spot picking, destaining, digestion, extraction, sample preparation and spotting on MALDI target plates were carried out using a spothandling workstation (ETTAN Spothandling workstation, GE Healthcare) and a standard protocol provided by GE Healthcare. The plate containing the combined extracts was evaporated to dryness. Each sample was prepared by constituting the dried peptides in 2.5 µl of matrix solution (2.5 mg/ml of α-cyano-4-hydroxy-cinnamic acid (Sigma) in 50% acetonitrile containing 0.05% TFA). 2.0 µl sample was spotted on a clean MALDI target slide surface and allowed to dry. The samples were analysed with a vMALDI-LTQ (Thermo Electron, San José, CA, USA). The analysis was done using Xcalibur 1.4 software in data dependent mode. A survey scan (MS) was followed by MS/MS scans on the 5 most abundant ions. This string of 6 scan events was repeated six times for each sample spot. Dynamic Exclusion™ ensured that in total 30 different peptides were selected and fragmented for each sample. The MS spectra were collected in the 900–2000 Da mass range while the mass range for the MS/MS spectra were automatically selected by the system based on a Q value of 0.25. The standard collision energy of 38 was set for all the analysis. A time limit of 5 minutes/sample was selected, whether or not the 30 MS/MS spectra could be acquired. Database searches were done using both the MASCOT and Sequest search algorithm against the human session of the IPI protein database (version 2.38). The two searches were compared in the in house developed software Promiscuous MS/MS. A minimum of two peptides and A Mascot score of 45 were required for a protein to be accepted as identified.

## Results

### Establishment of androgen-independent cell line, LNCaP-s and detection of AR, CgA and NSE expression in LNCaP-s cells

To address the natural progression of prostate cancer from androgen sensitive to androgen independent state, a prostate cancer cell model is very important for *in vitro* study. So we cultured a LNCaP-s cell line from a parental prostate cancer cell line LNCaP in a androgen-deprivation condition. NE cells are characterized by a neuronal-like phenotype which produce and secrete a series of neuropeptides involved in tumor proliferation, transformation and metastasis [19]. The morphologic characteristics showed a neuronal morphology with compactly rounded cell bodies, having extended and fine branched processes. Thus androgen-sensitive LNCaP cells acquired a NE-like phenotype (Figure 1) LNCaP-s in an androgen-reducing condition. The NE-like cells, characteristics were evaluated by testing the markers of NED, chromogranin A (CgA) and neuron-specific enolase (NSE). After culturing in the androgen-reduced condition, the LNCaP cells showed a decreased expression level of AR, an increased NSE expression level, but CgA with no significant expression. Figure 1 showed different expressions of AR, CgA and NSE in LNCaP-s cells.

**Figure 1:** Characterizition of LNCaP-s cells. Parental LNCaP cells have an epitheial morphology and LNCaP-s cells showed a neuronal morphology. AR, CgA and NSE expressions in LNCaP and LNCaP-s cells examined by RT-PCR and Western Blotting.

### smsDX inhibited the invasiveness of prostate cancer cells

It is well established that somatostatin and its analogue effects on the proliferation of prostate cancer cells [20]. But the somatostatin effects on invasiveness had not been investigated. To assess the effects of smsDX on the invasiveness of prostate cancer cells we used wound healing assay and Matrigel™ invasion assay, The covered area in the wound and the number of cells invading through a Matrigel chamber were significantly smaller for cells treated with smsDX than they were for control cells treated with vehicle in LNCaP and LNCaP-s cells (Figure 2 and 3). The inhibition of smsDX shows a dose-dependent manner with the cell number invading ability in both LNCaP and LNCaP-s cells. These results suggest that smsDX decreased the invasiveness of prostate cancer cells.

**Figure 2:** Inhibition of cell migration of prostate cancer cells LNCaP/LNCaP-s by smsDX. Representative photomicrographs demonstrate wound closure in LNCaP cells (A) and LNCaP-s cells (B). Monolayers of LNCaP/LNCaP-s cells were disrupted with sterile pipette tip to create uniformand treated with PBS or 1–10 nM smsDX for 24 hours.

**Figure 3:** Inhibition of cell invasiveness of prostate cancer cells LNCaP/LNCaP-s by smsDX. Matrigel invasion data when LNCap/LNCaP-s cells in upper well were incubated in serum-free medium and lower well was filled with serum-free medium and 1–10 nM smsDX or PBS. After 24 hours, number of cells that invaded through Matrigel was counted in at least 10 fields per well. Representative photographs reveal LNCaP (A) and LNCaP-s (B) cells that invaded through Matrigel. Reduced from ×100.

### 2D gel electrophoresis analysis

Figure 4 shows representative 2D gels of control and smsDX samples in LNCaP and LNCaP-s cells. Three replicates were run for each group, control and smsDX. The smsDX effects on LNCaP and LNCaP-s cells were compared separately with the control group using a Mann-Whitney test.

**Figure 4:** Representative examples of 2-DE gels. Whole-cell lysate was subjected to 2-DE using IPG strips pH 3–10 in the first and 12.5% SDS polyacrylamide gel in the second dimension. A, Parental LNCaP cells, B, derivative LNCaP-s cells. C, LNCaP+smsDX , D, LNCaP-s+smsDX.

### Proteins differentially expressed between LNCaP and LNCaP-s cells

A total of 222 spots were successfully identified using 2DE-based MS. In the first analysis, smsDX-treated LNCaP cells were compared to LNCaP control group using a Mann-Whitney test. 56 proteins were found to be differentially expressed in LNCaP and LNCaP-s (Table S1). In the second analysis, 104 and 86 proteins, separately, were found differentially expressed in LNCaP cells and LNCaP-s cells following smsDX treatment (Table S2A and Table S2B). The expression of specific isoforms of metabolic enzymes has been showed to be crucial for the adaptation of tumor cells to changes in nutrient availability, especially for glycolytic enzymes [21]. So isoforms of proteins were also listed in this table. The same protein was sometimes found in multiple closing spots on 2DE gels, it is possible due to posttranslational modification of protein after stress.

Fifty-six proteins were found down-expressed (more than 1.2-fold change) in LNCaP-s cells compared to the parental LNCaP cells, as listed in table S1.

Proteins both in LNCaP and LNCaP-s cells affected by smsDX incubation with a fold change ≥1.2 were listed in table S2A and table S2B.

### Sorted functions of proteins in the effect of smsDX on prostate cancer (LNCaP-s) cells after ADT treatment

The different functions of proteins with accession code refer to the website, http://www.uniprot.org/uniprot/. The proteins identified were categorized on the basis of their known biochemical functions including metabolism, signalling transduction, maintenance of cell structure, transcriptional regulation and cell cycle regulation. Most of androgen deprivation stressed proteins were down-regulated after ADT treatment. When we explored these protein functions within the website UniProtKB/Swiss-Prot, surprisingly, most of the proteins affected by ADT therapy were found to be involved in the cell metabolism and mitochondrial function regulation. Based on the putative functions in the KEGG pathway database (http://www.genome.jp/kegg/pathway.html), Table S3(A,B,C) were derived from table S2A and table S2B to highlight the similarities/differences in the effect of smsDX between LNCaP and LNCaP-s cell lines. Table S3A listed forty-eight common proteins between LNCaP and LNCaP-s cells after exposure to smsDX. Table S3B, S3C listed the differentially affected proteins in LNCaP and LNCaP-s cells, separately.

Androgen deprivation could affect mitochondrial protein expression, for example, HSPD1, ETFA, GLUD1, PMPCB and et al. These proteins were found belonging to mitochondrial proteins involving in glucose metabolism, the production of reactive oxygen species (ROS) and intrinsic mitochondrial-mediated apoptotic function. The proteins with important roles in cell metabolic process, including energy (APRT, ATP5B, CKB, TUBB), lipid (ACAT2, ACADM, PRDX6), glucose (ENO1, TPI1) and amino acid and protein biosynthesis (PHGDH, EIF5A, EIF1AY) , were found down-regulated in LNCaP-s cells. Some metabolic enzymes involved in the TCA were also identified. ADT treatment leads to a decline in the protein expression of several ER chaperones, including GRP78, ERP29, PDIA1 and PDIA3 protein.

### Validation of proteins affected by smsDX and ADT treatment in prostate cancer cells with Western Blotting

Proteins in LNCaP-s cells involving in different signaling pathways were identified in this current study, these proteins could be regulated by smsDX at different change fold as listed in table S2. Validation of proteins affected by smsDX and ADT treatment in prostate cancer cells were carried out by Western Blotting. Several mitochondrial proteins, ER proteins and proteins involving metabolism were selected to detect for validation with immunoblotting. Figure 5 showed that TCTP, STMN1, and CXB3 in LNCaP cells after ADT were down-regulated and TOM40, GRP78 and VDAC2 which involving in the mitochondrial activity in LNCaP-s cells were up-regulated by when treated with smsDX.

**Figure 5:** Validation of selected proteins by using western blotting. A, Lower expressions of protein TCTP, STMN1, and CXB3 in LNCaP cells after ADT in LNCaP-s cells. B, Down regulated expressions of TOM40, GRP78 and VDAC2 in LNCaP cells by androgen-deprivation, up regulated expressions in LNCaP-s cells by smsDX treatment.

### Metabolic pathways regulated by somatostatin derivative (smsDX) in prostate cancer cells

Based on the KEGG pathway database (http://www.genome.jp/kegg/pathway.html), we presented a diagram of metabolic pathways regulated by smsDX in prostate cancer from androgen dependent to CRPC status (Figure 6). The enzymes in circle were identified by 2-DE MS in this current study.

**Figure 6:** Metabolic pathways regulated by somatostatin dervivative (smsDX) in prostate cancer cells. Enzymes and metabolites that are part of glycosis, fatty acide synthesis and the TCA cycle are shown. G6PD, Glucose-6-phosphate 1-dehydrogenase. ENO1, Alpha enolase. PPP, pentose phosphate pathway. ACAT2, Acetyl-CoA acetyltransferase. ACAMD, Acyl-CoA dehydrogenase. IDH2, Isocitrate dehydrogenase [NADP]. MDHM, Malate dehydrogenase. GLUD1, Glutamate dehydrogenase1. α-KG, α-Ketoglutarate. This simplified diagram is based on the KEGG pathway database (http://www.genome.jp/kegg/pathway.html). The enzymes in circle were identified by 2-DE MS in this current study.

## Discussion

Androgen plays an essential role in prostate cancer growth, so androgen deprivation and the blockade of AR signaling axis is currently the main treatment for prostate cancer and its progression. It is well documented that clinical androgen-deprivation therapy is associated with increased NE differentiation in prostate carcinomas, and involved in the transition to androgen independence [22], NE cells are characterized by a neuronal-like phenotype: they are non-proliferative and express neuronal-like proteins, such as NSE and CgA. Androgen deprivation can influence the serum CgA levels to different extents in prostate cancer [23]. The overexpression of NSE in LNCaP-s in our study was found in the progression of NED from androgen dependent LNCaP cells. In this current study, after up to 10 passages of LNCaP cells in a reduced androgen condition, the NE-like characteristics of LNCaP-s were identified by a neuronal morphology and altered expressions of AR and NSE.

The effects of somatostatin inhibition on cancer cell viability and proliferation have been well examined but to our knowledge, its effects on invasiveness had not been investigated. Using wound healing and Matrigel invasion assay we observed that smsDX inhibited the invasiveness of both LNCaP and LNCaP-s cells. Although the exact mechanisms of smsDX induced suppression of invasiveness are not currently clear, it might be due to responses to damaged mitochondrial functions. In our previous studies [7], [24], smsDX regulated mitochondrial and related proteins both in androgen dependent and independent prostate cancer cells, so the cancer-associated alterations in metabolism are possibly responsible for the cell proliferation and survival signals in recurrent prostate cancer and CRPC.

To determine the metabolism regulation effects of smsDX on progression of prostate cancer from androgen-dependent to androgen independent status, we performed two-dimensional gel electrophoresis (2-DE) followed by MALDI-TOF mass spectrometric analysis. After comparison of protein expression in LNCaP-s and its parental LNCaP cells, fifty-six proteins were found to be differentially expressed up to 1.2 fold change as showed in table S1. These proteins were sorted according to their different functions in cell metabolism, including sugar, energy, lipid and amino acid process. The results suggest that androgen-regulated metabolic alteration is the main differences during the development of prostate cancer from androgen-sensitive to androgen-resistant status. The similar and different effects caused by smsDX were found between LNCaP and LNCaP-s cells. The stress caused by androgen deprivation and smsDX to prostate cancer cell environment could possibly caused mitochondrial function damage and activate AMPK pathway in the prostate cancer cells. Mitochondrial processes play an important role in tumor initiation and progression. Increased metabolic activity is a hallmark of proliferating cancer cells [25]. So suppressing the cancer cell metabolic activity provides an alternative strategy for CRPC stage. ADT for prostate cancer caused abnormal microenvironment condition elicit responses from tumor cell to affect metabolic activity. These adaptations optimize tumor cell metabolism to get energy and nutrients from tumor microenvironment. Several reports have shown that androgen biosynthesis and AR signaling in prostate cancer cells are intimately affected by lipogenesis [26]–[28]. So targeting the possible underlying molecular mechanisms linking metabolism could facilitate further development of promising therapeutic approaches for CRPC status.

Based on the data we collected here, we found the smsDX regulated PI3K/AKt/mTORC1 pathway and TCA cycle via up and down regulating different metabolic proteins listed in tbale S2A and table S2B. In prostate cancer AKt is activated via the PI3K pathway that has emerged as a critical pathway for cell survival. Removing androgen support from LNCaP cells triggers a series of events, including cell cycle arrest and increased PI3K/Akt activity, culminating in the eventual acquisition of the androgen- independent phenotype [29]. Activated PI3K/AKt leads to enhanced glucose uptake and glycolysis [30].This pathway also promotes glucose carbon flux into biosynthetic pathways that rely upon functional mitochondrial metabolism, including fatty acid, cholesterol and isopronoid synthesis all require acetyl-CoA. AKt also activates ATP-citratelyase (ACL) promoting the conversion of mitochondrial-derived citrate to acetyl-CoA for lipid synthesis. mTORC1 is a well-characterized cell growth regulator acting as downstream of PI3K/AKt, has many effects interwined with mitochondrial metabolism. mTORC1 is best known for enhancing protein synthesis [25]. Alpha enolase (ENO1), also known as pyruvate dehydrogenase phosphatase, it is critical for cellular energy metabolism [31]. ENO1, as a key glycolytic enzyme, plays a critical role in anaerobic glycolysis. In this current study, ENO1 could be up regulated by smsDX, which showed that smsDX has a regulatory effect on glycolysis in prostate cancer cells.

The TCA cycle is a central pathway in the metabolism of sugars, lipids and amino acid, TCA cycle metablites result in reduced cellular differentiation. [32] Glutamine is a non-essential amino acid that is metabolized to glutamate and enters the TCA cycle as alpha-ketoglutarate, resulting in high ATP generation via oxidative phosphorylation [33]. Glutamine is the primary mitochondrial substrate and is required to maintain mitochondrial membrane potential and integrity as well as support of the NADPH production needed for redox control and macromolecular synthesis [34]. Mitochondrial enzyme glutaminase converted glutamine→glutamate→α-ketoglutarate (α-KG) by glutamate dehydrogenase, α-KG involves in TCA and can provide carbon backbones for cellular anabolic reaction [35]. NADPH functions as a cofactor and critical antioxidant provides the reducing power for both the glutathione (GSH) and thioredoxin (TRX) that scavenge ROS and repair ROS-induced damage [36]. NADP-dependent isocitrate dehydrogenase IDH1 and IDH2 convert isocitrate to α-KG. The metabolism of amino acid and fatty acids, like glucose, is reprogrammed to provide the building block for cancer cell growth and proliferation. DJ-1 and SOD1 identified in the current study were also found to have antioxidant properties [37]. Apparently, enzymes affected by smsDX, for example, glutamate dehydrogenase1, isocitrate dehydrogenase, glutathione synthetase, isocitrate dehydrogenase [NADP], Glucose-6-phosphate 1-dehydrogenase, were involved in the regulation of prostate cancer cell metabolism via different metabolic pathways. These adaptations altered tumor cell metabolism for proliferation by regulating multiple levels of energy in the form of ATP, biosynthetic capacity and the maintenance of balanced redox status. Here we demonstrated a simplified regulatory pathways (Figure 6) [38], [39] altered by smsDX during the development of prostate cancer. These metabolites and enzymes in this diagram, identified by 2-DE based MS analysis, are involving in the multiple pathways supporting cancer cells: glycolysis, TCA cycle, pentose phosphate pathway, glutaminolysis and lipid and nucleotide synthesis. For example, the acetyl-CoA groups (ACAT, ACADM and ACDSB) identified in our study could be activated by smsDX treatment which means the perturbation effect of smsDX on TCA cycle in mitochondrion in prostate cancer cells. Acetyl-CoA, a central metabolite at the intersection of carbohydrate, fatty acid, and acid oxidation, exerts tremendous influence on cell signaling.

Currently, very little information is currently available on the mitochondrial and ER proteins expression linked profile of clinical prostate cancer. The ER and mitochondria are physically and functionally linked, and there is increasing evidence of the GRPs influencing ER and mitochondrial cross-talk to maintain mitochondrial function. GRP78 is traditionally regarded as a major ER (endoplasmic reticulum) chaperone facilitating protein folding and assembly, protein quality control and regulating ER stress signaling [40]. The cytoplasmic GRP78 isoform is a newly identified regulator of the ER stress signalling pathway [41], in addition to the function of canonical GRP78 in the cytoplasm. Beyond the ER, the mitochondrial, nuclear and secreted forms of GRP78 have been linked to cellular homoeostasis and therapeutic resistance. The partial reduction in GRP78 in white adipose tissue leads to the elevated expression of GRP75, suggesting increased energy expenditure in the mitochondria probably as a compensatory measure. It is possible that GRP78 might physically interact with GRP75 in the mitochondria, since it has been reported that GRP78 is also localized in the mitochondria under ER stress [42]. GRP78 is expressed on the cell surface of prostate cancer cells and appears to mediate the signal transduction of Beta2-M [43]. It correlates with the development of androgen-independent disease and shorter overall survival in prostate cancer patients [44]. As a receptor, ligation of surface GRP78 with its ligands, such as α2-M and GRP78 auto-Abs, also activates the PI3K/Akt pathway. The activated PI3K/Akt pathway can further enhance the stability of GRP78 [45]. Thus, GRP78 and PI3K/Akt pathway may thereby constitute a positive feedback loop, which is involved in protecting tumors against hypoxia and nutrient starvation and regulating cell metabolism in the microenvironment. Arap et al. [46] has recently identified GRP78 as a potential molecular target that may prove useful for translation into clinical applications.

Our data show that: (i) proteins analysis of human prostate cancer cell lines reveals that proteins involving cancer cell metabolism could be alerted by smsDX. (ii) LNCaP-s was a derivative cell line from LNCaP cell lines, so it has the most same characteristics with LNCaP cells. After ADT treatment, most prostate cancer cells will die from starvation/energy stress, LNCaP cells become to LNCaP-s cells with NE-like phenotype which mimic the clinical progression from androgen dependent to androgen independent CRPC stage. Data presented in this article are collected from the study of established AR-positive, androgen-dependent and lower AR expression human prostate cancer cells (LNCaP/LNCaP-s), additional study may be warranted to define the links with the host microenvironment, for example, cancer-associated fibroblast cell interaction which was proposed by Sotgia F in his “two-compartment tumor metabolism” model, these catabolic host cells could fuel anabolic cancer cell growth and metastasis via mitochondrial metabolism. A study by Nieman KM et al., [47] shows that triglyceride catabolism in adipocytes drives ovarian cancer metastasis by providing fatty acids as mitochondrial fuels. In CRPC, however, somatostatin analogues were found ineffective when given as monotherapy. More promising results were obtained when lanreotide or octreotide were administered in combination with other agents within a novel concept of “antisurvival factor therapy” [48]. This concept aims to target not only the neoplastic cells but also various factors secreted in their microenvironment that confer protection from apoptosis. The combination of ethinyl estradiol and somatostatin analogue lanreotide offered a median overall survival that was superior to the 10-month median survival in patients with hormone refractory disease [23].

SmsDX could regulate the different metabolic enzymes and proteins which involving metabolic pathways supporting cancer cells: glycolysis, TCA cycle, pentose phosphate, glutaminolysis and oxidative phosphorylation in LNCaP-s cells. So we speculate that inhibition of invasiveness of LNCaP-s is possible due to regulation of metabolism of prostate cancer cells. So it's tempting to speculate the possible role of smsDX in the treatment of CRPC, but the complex crosstalk at multiple levels among them were not fully understood, so further validating investigations are needed.

Taken together, alterations of AR affected by androgen-deprivation could change prostate cancer cell metabolism via multiple intra- and extra-cellular signaling pathways, smsDX effects on the cancer cell metabolism regulating energy, lipid, amino acid and protein biosynthesis provide in-depth information to improve the response to therapy and result in a positive clinical outcomes. The smsDX targeting effects on cellular metabolism in androgen-dependent prostate cancer after ADT therapy improve our understanding of somatostatin's anti-cancer mechanism(s) and possibly lead to the introduction of a novel therapeutic approach for CRPC.

## Supporting Information

Table S1 **Fifty -six lower expressed proteins in LNCaP-s compared to LNCaP cells (≥1.2 in fold change).** LNCaP cells were cultured from androgen-sensitive LNCaP parental cells, in an androgen-reduced condition. Proteins of the parental LNCaP cells after ADT were identified by means of two-dimensional gel electrophoresis (2-DE) followed by MALDI-TOF mass spectrometric analysis.
(XLSX)

Table S2 **Proteins affected by smsDX incubation with a fold change ≥1.2 both in LNCaP (table S2A) and LNCaP-s (table S2B) cells.** Protein accession numbers from SwissProt/TrEMBL are given and “trend” indicates the direction of the change in expression level. Ctrl: control, SD: smsDX.
(XLS)

Table S3 **Proteins highlighting the similarities/differences in the effect of smsDX between LNCaP and LNCaP-s cell lines.** Sorted function descriptions were included in these tables. Table S3A listed forty-eight common proteins between LNCaP and LNCaP-s cells after exposure to smsDX. Table S3B, S3C listed the differentially affected proteins in LNCaP and LNCaP-s cells, separately. Proteins with mark#indicate the common proteins in Table S1.
(XLS)
